RETRACTED

# Kinetin mitigates Cd-induced damagesto growth, photosynthesis and PS II photochemistry of *Trigonella* seedlings by up-regulating ascorbate-glutathione cycle

**DOI:** 10.1371/journal.pone.0249230

**Published:** 2021-06-22

**Authors:** Gausiya Bashri, Shikha Singh, Sheo Mohan Prasad, Mohammad Javed Ansari, Salma Usmani, Saleh Alfarraj, Sulaiman Ali Alharbi, Marian Brestic

**Affiliations:** 1 Department of Botany, Ranjan Plant Physiology and Biochemistry Laboratory, University of Allahabad, Allahabad, India; 2 Department of Botany, Hindu College Moradabad, Mahatma Jyotiba Phule Rohilkhand University, Bareilly, India; 3 Department of Biochemistry, D.K.M College for Women (Autonomous), Vellore, India; 4 Zoology Department, College of Science, King Saud University, Riyadh, Saudi Arabia; 5 Department of Botany & Microbiology, College of Science, King Saud University, Riyadh, Saudi Arabia; 6 Department of Plant Physiology, Slovak University of Agriculture, Nitra, Slovakia; Harran Üniversitesi: Harran Universitesi, TURKEY

## Abstract

Cytokinins (CKs) plays a key role in plant adaptation over a range of different stress conditions. Here, we analyze the effects of a cytokinin (i.e., kinetin, KN) on the growth, photosynthesis (rate of O_2_ evolution), PS II photochemistry and AsA–GSH cycle in *Trigonella* seedlings grown under cadmium (Cd) stress. *Trigonella* seeds were sown in soil amended with 0, 3 and 9 mg Cd kg^-1^ soil, and after 15 days resultant seedlings were sprayed with three doses of KN, i.e.,10 μM (low, KN_L_), 50 μM (medium, KN^M^) and 100 μM (high, KN_H_); subsequent experiments were performed after 15 days of KN application, i.e., 30 days after sowing. Cadmium toxicity induced oxidative damage as shown by decreased seedling growth and photosynthetic pigment production (Chl *a*, Chl *b* and Car), rates of O_2-_evolution, and photochemistry of PS II of *Trigonella* seedlings, all accompanied by an increase in H_2_O_2_ accumulation. Supplementation with doses of KN at KN_L_ and KN_M_ significantly improved the growth and photosynthetic activity by reducing H_2_O_2_ accumulation through the up-regulation AsA–GSH cycle. Notably, KN_L_ and KN^M^ doses stimulated the rate of enzyme activities of APX, GR and DHAR, involved in the AsA–GSH cycle thereby efficiently regulates the level of AsA and GSH in *Trigonella* grown under Cd stress. The study concludes that KN can mitigate the damaging effects of Cd stress on plant growth by maintaining the redox status (>ratios: AsA/DHA and GSH/GSSG) of cells through the regulation of AsA-GSH cycle at 10 and 50 μM KN under Cd stress conditions. At 100 μM KN, the down-regulation of AsA-GSH cycle did not support the growth and PS II activity of the test seedlings.

RETRACTED

## Introduction

Contamination of air, soil and water due to various kinds of pollutants which are byproduct of industrial activity has created a worldwide problem [1–3]. In recent years, heavy metals are the most important contaminants causing serious threat to the life of every living being. Cadmium (Cd) is considered the most toxic of such pollutant metals because of its rapid uptake and translocation, combined with its ability to bind sulphahydryl group of enzymes/ proteins. Cadmium levels are increasing in agricultural soils due to the application of phosphate fertilizers and municipal Increased Cd inhibits plant growth by reducing photosynthesis by interfering with photosystem II (PS II) photochemistry, and by altering the leaf-ultrastructure, particularly that of chloroplasts [4]. A major mechanism of Cd- induced damage in plant is an increase in the generation of reactive oxygen species (ROS) due to disturbance of mitochondrion and chloroplast electron transport chain via the displacement of essential cations like Ca^2+^ and Zn^2+^ [5]. Increased generation of ROS, such as O_2_¯, H_2_O_2_, and HO¯ leads to oxidative stress by damaging the cell membranes through lipid peroxidation and proteins degradation, which results in disturbed cellular homeostasis [6, 7]. Plants protect themselves from ROS impairment through the mutual action of enzymatic and non-enzymatic antioxidants and the main pathway for scavenging of H_2_O_2_ is ascorbate (AsA)-glutathione (GSH) cycle [8, 9]. Here, the reduction of H_2_O_2_ into water is catalyzed by the enzyme ascorbate peroxidase (APX) with the help of AsA, which serve as an electronic donor. In addition, dehydroascorbic acid (DHA) is reduced by the enzyme dehydro ascorbate reductase (DHAR) by consuming the electrons provided by reduced glutathione (GSH) which oxidize into glutathione disulfide (GSSG). The reduction of GSSG into GSH is catalyzed by the enzyme glutathione reductase (GR). The AsA–GSH cycle is therefore crucial for maintaining the reductive environment in plant cells via the up-regulation of its enzymes under a variety of stress conditions [5, 9].

Plant growth regulators (PGRs) play crucial roles in the growth and development of the plants, by altering various important physiological and biochemical processes required by plants when exposed to heavy metal toxicity [10]. In recent years, many PGRs have been shown to ameliorate the negative impacts of heavy metal toxicity [5, 11]. Cytokinins (CKs) for example, take part in numerous physiological activities such as cell division and morphogenesis, flower and seed development and chloroplast development [12–16]. CKs can also regulate the abiotic stresses by the up-regulation of nitrogen metabolism and antioxidant defense system of plants [12, 17–21]; the importance of CKs in the regulation of heavy metal stress tolerance in plants is well known [11, 17, 18, 22], but the mechanism of CKs induced regulation of heavy metal stress tolerance needs further investigation. The work reported here aimed to determine the effect of exogenous application of different level of KN (KN_L_, KN_M_ and KN_H_) on *Trigonella* seedlings (in order to counteract Cd phyto-toxicity) by examining their effects on growth and photochemistry of the PS II and AsA–GSH cycles.

RETRACTED

## Material and methods

### Plant material and growth conditions

Seeds of *Trigonella foenum-graecum* L. var. Antara were procured from the Suttind seeds Pvt. Ltd, Delhi. The growth conditions used are the same as described by Bashri and Prasad [5]. The selected doses i.e. 3 mg Cd kg^-1^ soil (Cd_1_) and 9 mg Cd kg^-1^ soil (Cd_2_) of Cd were applied in the soil before seed-sowing. After 15 days of growth the seedlings were treated with three doses of KN, i.e., 10 μM (low, KN_L_), 50 μM (medium, KN_M_) and 100 μM (high, KN_H_) exogenously. The tested doses (KN_L_, KN_M_ and KN_H_) of KN were selected on the basis of screening experiment with 1, 5, 10, 25, 50, 75 and 100 μM of KN. The experimental scheme contains twelve combinations i.e. control, Cd_1_, Cd_2_, KN_L_, Cd_1_+KN_L_, Cd_2_+KN_L_, KN_M_, Cd_1_+KN_M_, Cd_2_+KN_M_, KN_H_, Cd_1_+KN_H_, Cd_2_+KN_H_. All experiments were performed following 15 days of KN application.

### Determination of growth, and pigments: Chlorophylls and carotenoids

Plant growth was analyzed by determining the fresh and dry weight, height and leaf area. Seedlings were harvested and their fresh weight was determined immediately; dry weight determination was achieved by drying the plant samples at 80°C for 48 h in hot air oven. The height of the plants was recorded by the meter scale. The leaf area of seedlings was analyzed by leaf area meter (Model—211, Systronics, India). For the estimation of pigments (chlorophylls and carotenoids), 20 mg fresh leaves were extracted with 80% (v/v) acetone and optical density of the supernatant was measured at 663.2, 646.5 and 470 nm spectrophotometrically [23].

### Determination of carbonic anhydrase (CA) activity and rates photosynthesis and respiration

The activity of CA in leaves was measured by the method of Wilbur and Anderson [24]. The rate of photosynthesis and respiration was estimated in leaf discs using a Clark type oxygen electrode in terms of O_2_ evolution / consumption in the presence and absence of light, respectively and expressed as μmol oxygen evolved / consumed g^-1^ FW h^-1^ [25].

RETRACTED

### Chlorophyll *a* fluorescence (PS II photochemistry) measurements

Different JIP (**JIP** is a dark adapted chlorophyll fluorescence technique that is used for plant stress measurement)-parameters i.e. φP_0_ or Phi_P_0_, Ψ_0_ or Psi_0, φE_0_ or Phi_E_0_, PI_ABS_, ABS/RC, TR_0_/RC, ET_0_/RC and DI_0_/RC of PS II photochemistry of control and treated seedlings were measured as chlorophyll *a* fluorescence through leaf fluorometer (FluorPen FP 100, Photon System Instrument, Czech Republic) in 30 minutes dark adapted leaves [26]. The values presented in the form of radar chart by normalizing all the data with their respective controls and control value for all parameters in radar chart is one.

### Determination of hydrogen peroxide (H_2_O_2_): *In vitro* and *in vivo* analysis

Hydrogen peroxide determination was performed using 40 mg fresh leaves, and the supernatant was obtained by homogenization of these leaves in 3 ml of 0.1% (w/v) trichloro acetic acid after centrifugation (10,000 g for 15 min). The method described by Velikova et al. [27] was used; the amount of H_2_O_2_ in each sample is expressed as nmol g^—1^ FW. The localization of H_2_O_2_ in leaves was determined using a 1% solution of 3, 3’-diaminobenzidine, and bleaching with boiling ethanol, then photographed by digital camera [28].

### Determination of activities of enzymes of ASC and GSH cycle

The activity of APX was determined by the method described by Nakano and Asada [18], with one unit of enzyme activity being defined as 1 nmol AsA oxidized min^-1^. Activity of DHAR was analyzed by extinction coefficient of 7.0 mM^−1^ cm^−1^; one unit of DHAR activity is defined as 1 nmol DHA reduced min^-1^ [29]. GR activity was estimated by extinction coefficient of 6.2 mM^-1^ cm^-1^; one unit of GR activity is defined as 1 nmol NADPH oxidized min ^-1^ [30].

### Determination of ascorbate and glutathione

Ascorbate content was determined as described by Gossett et al. [31]. The absorbance for ascorbate content was recorded at 525 nm and calculated using a standard curve prepared with L-ascorbic acid. Glutathione content was determined using the method described by Brehe and Burch [32] in a leaf homogenate, absorbance was recorded at 412 nm. Glutathione amount was then determined using a standard curve prepared with GSH.

### Statistical analysis

Data presented is the means of triplicate (n = 3). One-way ANOVA test was performed to test the significance of data which was carried out at P<0.05 significance level using Duncan’s multiple range test (DMRT).

## Results

### Effect of KN on growth and photosynthetic pigments under Cd stress

Cadmium treatments significantly (P<0.05) reduced plant fresh and dry weight with increasing Cd concentration (Fig 1). *Trigonella* seedlings grown under Cd_1_ and Cd_2_ stress showed decrease in both fresh weight (by 13 and 20%) and in dry weight (by 8 and 14%);the reduction in leaf area was 6 and 12%, respectively. Supplementation of KN_L_ (10 μM KN) significantly improved the repressing effects of Cd on growth, the effect being more pronounced under Cd_1_ stress.

RETRACTED

**Fig 1:** Impact of foliar application of kinetin on growth attributes of *Trigonella* seedlings exposed to Cd stress. Data represent the mean value ± standard error from three replicates (n = 3). Values followed by the different letters at each bar differ at P<0.05 among treatments by the DMRT.

Similarly, KN_M_ (50 μM KN) marginally alleviated the Cd toxicity in *Trigonella* seedlings. High dose of KN (KN_H_,100 μM KN), in contrast, increased the Cd induced toxicity showing the decline of 17 and 26% in fresh weight and 18 and 34% in dry weight exposed to Cd stress (Cd_1_ and Cd_2,_ respectively). Plant height also declined by 7 and 17% under Cd stress (Cd_1_ and Cd_2,_ respectively). Exogenous KN_L_ under the similar conditions, mitigated the Cd induced toxicity, the reduction being only 3 and 8% under Cd stress (Cd_1_ and Cd_2,_ respectively). In contrast, KN_H_ aggravate the Cd induced effect and the decline was 15 and 27%, respectively (Fig 1). Cadmium application at both doses significantly (P<0.05) decreased the Chl *a*, Chl *b* and Car contents in *Trigonella* seedlings. The exogenous application of kinetin at KN_L_ and KN_M_ doses in Cd treated seedlings resulted in a considerable reduction in all the pigment contents. On the other hand, KN_H_ application lead to an additional declined in Chl *a*, Chl *b* and Car contents of *Trigonella* seedlings exposed to Cd stress (Table 1).

**Table 1:** Effect of KN on photosynthetic pigment contents of *Trigonella* seedlings exposed to Cd stress.

Treatments	Pigment contents (mg g^—1^ FW)			Ratio	
	Chl *a*	Chl *b*	Car	Chl *a* / *b*	Total Chl*/* Car
Control	1.330±0.017^fg^	0.482±0.012^gh^	0.350±0.006^de^	2.777±0.071^a^	5.175±0.087^d^
Cd_1_	1.255±0.018^cd^	0.415±0.006^d^	0.330±0.004^bc^	3.022±0.040^cde^	5.062±0.071^bcd^
Cd_2_	1.150±0.016^ab^	0.375±0.004^ab^	0.305±0.004^a^	3.065±0.039^e^	5.003±0.087^bcd^
KN_L_	1.488±0.022^i^	0.510±0.013^i^	0.400±0.009^g^	2.918±0.105^bcd^	4.996±0.098^bcd^
Cd_1_ + KN_L_	1.373±0.020^gh^	0.490±0.007^h^	0.370±0.018^f^	2.803±0.042^ab^	5.036±0.270^bcd^
Cd_2_ + KN_L_	1.278±0.018^def^	0.440±0.007^e^	0.338±0.008^cd^	2.905±0.041^bc^	5.079±0.091^cd^
KN_M_	1.425±0.021^h^	0.487±0.015^h^	0.396±0.015^g^	2.928±0.087^bcd^	4.834±0.387^ab^
Cd_1_ + KN_M_	1.322±0.019^efg^	0.453±0.015^ef^	0.357±0.012^ef^	2.915±0.092^bdc^	4.977±0.309^bcd^
Cd_2_ + KN_M_	1.203±0.017^bc^	0.392±0.012^bc^	0.340±0.009^cd^	3.072±0.092^e^	4.691±0.242^a^
KN_H_	1.270±0.018^de^	0.464±0.009^fg^	0.333±0.005^bc^	2.739±0.053^a^	5.201±0.129^d^
Cd_1_ + KN_H_	1.233±0.018^cd^	0.405±0.008^cd^	0.320±0.005^b^	3.045±0.050^de^	5.122±0.114^cd^
Cd_2_ + KN_H_	1.132±0.016^a^	0.358±0.005^a^	0.303±0.004^a^	3.158±0.046^e^	4.912±0.071^abc^

Data represent the mean value ± standard error from three replicates (n = 3). Values followed by the different superscripts within same column differ at P<0.05 among the treatments by DMRT.

RETRACTED

### Effect of KN on CA activity, rate of photosynthesis and respiration under Cd stress

Cadmium toxicity decreased CA activity by 35 and 47% exposed to Cd stress (Cd_1_ and Cd_2,_ respectively). Exogenous supplementation of KN_L_ dose completely reinstated the CA activity at Cd_1_ dose while at Cd_2_ dose enhancement was recorded, showing only 5% decrease in CA activity. The application of KN_H_ further decreased the CA activity under Cd stress (Fig 2B). As with CA activity, the rate of photosynthesis was significantly (P<0.05) inhibited by Cd in *Trigonella* seedlings which showed a 16 and 24% decrease, respectively under Cd_1_ and Cd_2_ stress. Exogenous kinetin at KN_L_ and KN_M_ doses significantly ameliorated Cd-induced inhibition while KN_H_ treatment further inhibited the photosynthetic activity showing 24 and 29% reduction, respectively under Cd_1_ and Cd_2_ stress (Fig 2A). The respiratory activity was enhanced significantly under both the doses of Cd in leaves *Trigonella* seedlings, showing increases of 7 and 16%, respectively under Cd_1_ and Cd_2_ stress. The exogenous application of KN_L_ and KN_M_ doses considerably decreased the O_2_ uptake under Cd stress. On the other hand, KN_H_ dose supplementation resulted in an enhancement of 11 and 17% in the respiratory activity under Cd_1_ and Cd_2_ dose, respectively (Fig 2C).

**Fig 2:** Impact of foliar application of KN on photosynthetic O_2_ yield, carbonic anhydrase activity and respiration rate of *Trigonella* seedlings exposed to Cd stress. Data represent the mean value ± standard error from three replicates (n = 3). Values followed by the different letters at each bar differ at P<0.05 among treatments by the DMRT.

### Effect of KN on PS II photochemistry under Cd stress

The Photochemistry of PS II were analyzed in *Trigonella* seedlings exposed to Cd stress showed a marginal decrease in φP_0_ or Phi_P_0_, Ψ_0_ or Psi_0 φE_0_ at both the doses of Cd whereas PI_ABS_ declined significantly. Foliar application of KN_L_ and KN_M_ doses under Cd stress showed a significant alleviation in φP_0_, Ψ_0_, φE_0_ and PI_ABS_ however, with KN_H_ dose (Cd+KN_H_) the values of φP_0_, Ψ_0_, φE_0_ and PI_ABS_ were showing further reduction. Moreover, Cd stress enhanced the energy flux parameters i.e. ABS, TR_0_, ET_0_ and DI_0_ per RC (Fig 3). Kinetin application at KN_L_ and KN_M_ doses significantly reduced the energy flux parameters in *Trigonella* seedlings exposed to Cd stress. On the other hand, KN_H_ application caused a further increase in energy flux parameters (Fig 3).

RETRACTED

**Fig 3:** Impact of foliar application of KN on JIP—parameters in *Trigonella* seedlings exposed to Cd stress.

### Impact of KN on hydrogen peroxide level under Cd stress

Cadmium at Cd_1_ and Cd_2_ doses led to an increase in H_2_O_2_, by 28 and 67%, respectively. The exogenous application of KN at low and middle doses led to a significant (P<0.05) lowering in H_2_O_2_ content. In contrast, higher doses of KN (KN_H_) caused a further rise in H_2_O_2_ content over the values recorded in Cd_1_ and Cd_2_ treated seedlings (Fig 4A). The *in vivo* localization of H_2_O_2_ was performed with DAB. Cadmium treated seedlings showed a significant accumulation of brown precipitate as compared to the control which depends upon H_2_O_2_ content. Brown precipitates were less intense in the low and middle doses of KN treated *Trigonella* seedlings under Cd stress, indicating that H_2_O_2_ accumulation was lower in exogenously treated KN_L_ and KN_M_ seedlings. In contrast, higher dose (KN_H_) alone and together with Cd stressed seedlings exhibited a more intense brown color in leaf than that seen in the respective control (Fig 4B).

**Fig 4:** Impact of foliar application of KN on *in—vivo* localization of hydrogen peroxide in *Trigonella* seedlings exposed to Cd stress. *Trigonella* leaves stained with DAB, and brown area shows hydrogen peroxide content.

### Impact of KN on AsA-GSH cycle under Cd stress

Cadmium treatments at both the doses significantly (p<0.05) increased the activities of APX, DHAR (except at Cd_2_) and GR. The exogenous application of KN at low and middle doses further increased the rate of activity of these enzymes exposed to Cd stress; and these effects being most pronounced following KN_L_ treatments. The application of KN_H_ under Cd treatment showed variable responses (Fig 5). Cadmium stress caused a significant decrease in contents of AsA and GSH while the contents of DHA and GSSG were increased that result in sharp decrease in the ratios of AsA/DHA and GSH/GSSG. The exogenous application of KN at low (KN_L_) and middle (KN_M_) doses increased AsA and GSH and decreased DHA and GSSH as a result of this ratios of AsA/DHA and GSH/GSSG significantly increased in Cd-exposed seedlings; KN_H_ application resulted in opposite trends in the contents of AsA, DHA, GSH, GSSG and the ratios of AsA/DHA and GSH/GSSG (Table 2).

RETRACTED

**Fig 5:** Impact of foliar application of KN on ascorbate peroxidase, dehydroascorbate reductase and glutathione reductase activities of *Trigonella* seedlings exposed to Cd stress. Data represent the mean value ± standard error from three replicates (n = 3). Values followed by the different letters at each bar differ at P<0.05 among treatments by the DMRT.

**Table 2:** Impact of KN on the contents of reduced asorbate (AsA), dehydroascorbate (DHA), reduced glutathione (GSH), and oxidized glutathione (GSSG), and ratios of AsA/DHA and GSH/GSSG in *Trigonella* seedlings exposed to Cd stress.

Treatments	Contents (nmol g^—1^ FW)				Ratio	
	AsA	DHA	GSH	GSSG	AsA/DHA	GSH/GSSG
Control	830.00±11.98^e^	569.50±8.22^c^	225.82±3.25^g^	141.14±2.03^a^	1.45±0.025^e^	1.60±0.027^j^
Cd_1_	733.00±10.58^c^	612.50±8.83^de^	150.55±2.17^c^	207.00±2.98^d^	1.20±0.020^c^	0.73±0.012^d^
Cd_2_	603.00±8.704^a^	696.50±10.05^g^	117.68±1.70^b^	229.33±3.31^f^	0.86±0.015^a^	0.51±0.004^b^
KN_L_	989.25±14.27^g^	500.50±7.22^a^	301.69±4.35^j^	135.14±2.03^a^	1.98±0.031^h^	2.23±0.035^l^
Cd_1_ + KN_L_	878.90±12.68^f^	551.32±7.95^bc^	235.31±3.39^h^	168.78±2.58^c^	1.59±0.025^f^	1.39±0.020^i^
Cd_2_ + KN_L_	802.50±11.58^de^	611.00±8.81^de^	187.35±2.70^e^	208.42±3.12^d^	1.31±0.019^d^	0.90±0.014^f^
KN_M_	901.23±13.00^f^	531.50±7.67^b^	255.00±3.68^i^	138.62±2.17^a^	1.69±0.031^g^	1.84±0.035^k^
Cd_1_ + KN_M_	812.75±11.73^de^	614.00±8.86^de^	221.97±3.20^g^	165.73±2.62^c^	1.32±0.025^d^	1.34±0.020^h^
Cd_2_ + KN_M_	721.00±10.04^bc^	666.00±9.61^f^	171.74±2.48^d^	211.82±3.05^d^	1.08±0.019^b^	0.81±0.014^e^
KN_H_	787.50±11.36^d^	601.50±8.68^d^	198.33±2.86^f^	155.00±2.23^b^	1.31±0.021^d^	1.28±0.014^g^
Cd_1_ + KN_H_	692.50±9.99^b^	631.43±9.11^e^	142.73±2.06^c^	220.23±3.17^e^	1.09±0.017^b^	0.64±0.009^c^
Cd_2_ + KN_H_	595.00±8.58^a^	725.00±10.46^h^	77.29±1.11^a^	259.49±3.74^g^	0.82±0.025^a^	0.30±0.027^a^

Data represent the mean value ± standard error from three replicates (n = 3). Values followed by the different superscripts within same column differ at P<0.05 among the treatments by DMRT.

## Discussion

In present study, cadmium (Cd_1_ and Cd_2_) inhibited the growth of *Trigonella* seedlings, as shown by decreased plant height, leaf area and fresh and dry weight (Fig 1). The exogenous application of KN at KN_L_ (10 μM) and KN_M_ (50 μM) improved growth under Cd stress and the effect of KN_L_ (10 μM) being more pronounced. In consistent with our results, Zhou et al. [33] also reported better growth on exogenous application of cytokinin *trans*-zeatine riboside (10 μM) in *Kosteletzkyapenta carpos* under Zn stress. The observed KN-induced abatement of Cd toxicity on growth may be due to a decrease in Cd content in the plant as reported in earlier studies of eggplant [17]. In contrast to KN_L_ and KN_M_, KN_H_ application aggravates Cd-induced toxicity. This may be explained on the basis of excess accumulation of ROS and less efficient antioxidant system.

RETRACTED

Since the growth of autotroph depends on photosynthesis; hence the negative impact on growth of Cd stress can be correlated with an alteration in photosynthesis. Cadmium at both the doses decreased photosynthetic pigments (Chl *a*, Chl *b* and Car), a result which agrees with the findings of Ahanger et al. [18], in which Cd was shown to repress chlorophyll biosynthesis. The ameliorating effect of KN on photosynthetic pigment content could result from the regulatory effects of cytokinins on the biogenesis of chloroplast, as observedn wheat plants exposed to drought stress [34]. Further, cytokinins have been shown to stimulate the tetrapyrrole synthesis, hence supported the functioning of chloroplast in barley seedlings [35]. Another possibility could be due to decrease in reactive oxygen species like H_2_O_2_ (Fig 4) which is known to induce damaging effects on these pigments following Cd exposure under KN treatment. In contrast, the further degradation in pigment content seen in test seedlings treated with high doses of (KN_H_) of KN may be explained on the basis of excess accumulation of ROS (Fig 4) which probably triggered the degradation process at a greater rate under Cd stress. Photosynthetic oxygen yield during light reaction showed a direct link with photo-fixation of CO_2_ during Calvin cycle, hence Cd induced decrease in O_2_ yield in *Trigonella* seedlings, which leads to a decline in plant biomass accumulation, as observed in the present study (Fig 1). Popova et al. [36] reported that the exposure of pea plants to Cd at early stages of their establishment caused a decrease in the rate of CO_2_ fixation and the activity of Rubisco in the pea leaves. The significant improvement in photosynthetic activity seen in KN treated seedlings could be explained on the basis of (i) rise in light harvesting pigments i.e. Chl *a*, Chl *b* and Car contents (Table 1) and (ii) improved PS II activity as indicated by chlorophyll fluorescence activity (Fig 3). Aldesuquy et al. [34] reported that KN pre-treated wheat plant showed significant increase in the PS II activity and under salt stress; KN also ameliorated the PS II activity appreciably. Cadmium declined the activity of CA in test seedlings which might have resulted following the down regulation of genes for CA, as has been reported in *Populus tremula* under Cd stress [37]. It is also possible that Cd treatment may reduce Zn transport across the cell membrane, as Cd enters the cell via a Zn transporter protein [38]. Thus, decrease in Zn concentration in the leaf tissue may be one of the causes of decreased CA activity seen in the present study. *Trigonella* seedlings treated with low and middle doses of KN showed significant (P<0.05) improvement in CA activity under Cd stress. Fariduddin et al. [39] have similarly reported that KN and brassinosteroid treatment increased CA activity in *Vigna radiata*. The rate of O_2_ uptake was significantly increased by exposure to both doses of Cd, which can be explained on the basis of supply of ATP needed to carry out basic metabolism of plants, following a possible increase in rate of respiratory electron transport [40]. Cadmium treated seedlings on KN exposure exhibited a lower increase in rate of O_2_ uptake (Fig 2C). Al-Hakimi [41] also observed KN-induced decrease in respiration rate during Cd-stress in pea seedlings. To further validate the action of Cd on PS II, the photochemistry of PS II was analyzed in *Trigonella* seedlings exposed to Cd stress. Decrease in the values of φP_0_, Ψ_0_, φE_0_ and PI_ABS_ on treatment with the Cd (Fig 3) showing the inactivation of PS II and these results are in consistent with the earlier report on *Pontederia cordata* [4]. Further, Cd-induced increase in ABS/RC, TR_0_/RC, ET_0_/RC and DI_0_/RC could be explained on the basis of inactivation of active RC might be due to greater dissipation of flux [42]. KN induced improvements in JIP parameters under Cd exposure could be correlated with (i) anti senescing effect of KN, (ii) restoration in the status of D1 protein by increasing the antioxidants (Fig 5 and Table 2), as reported in cytokinin enriched *Arabidopsis* seedlings exposed to light stress [43], (iii) increased number of active RC (Fig 3). Tarakhovskaya et al. [44] also reported that KN increases the structural elements of Chl *a* including the PS II RC.

RETRACTED

In the present study, an over accumulation of H_2_O_2_ was observed following cadmium treatment (Fig 4) which points towards the oxidative stress induced by Cd [17, 18]. However, kinetin application, at low and medium concentration declined the level of H_2_O_2_, under Cd stress. In another study, kinetin treatment has been shown to improve the growth of root and shoot of maize seedlings, while it decreased the electrolyte leakage from leaf discs under Zn and Ni stress [45]. To remove the excess level of H_2_O_2_, one of the major mechanisms is AsA-GSH cycle. Although, Cd treatments increased the activities of APX, DHAR (except at Cd_2_) and GR but this increase was not sufficient for curtailing oxidative damage as evident with decreased growth (Fig 1). The exogenous application of KN at low and middle doses further enhanced the activity of APX, DHAR and GR in *Trigonella* seedling under Cd stress (Fig 5), suggesting the detoxification of H_2_O_2_ via AsA-metabolizing pathways by enzyme up-regulation. Cadmium stress caused significant decline in the contents of AsA and GSH and ratios of AsA/DHA and GSH/GSSG. The decrease in the level of AsA and GSH contents might be resulted due to their utilization in AsA-GSH cycle as electron donors and in synthesis of phytochelatins (particularly GSH) for metal detoxification. The exogenous application of KN at low (KN_L_) and middle (KN_M_) doses improved the AsA and GSH contents and declined the DHA and GSSG contents, resulting in increased ratios of AsA/DHA and GSH/GSSG in Cd exposed seedlings this may help *Trigonella* seedlings to preserve redox status under Cd stress. Wu et al. [46] also observed a BAP-induced increase of AsA and GSH contents under Zn stress. The application of KN_H_ under Cd treatment showed a variable response (Fig 5). In addition, glutathione synthetase and GR maintained the level of GSH, which ise involved in the biosynthesis and recycling pathways of GSH, respectively [8]. In the present work, a KN-induced increase of GSH content within the Cd-treated plants suggests that KN alters the regeneration of the GSH pool by stimulating GR enzyme. Our findings agree with those of Piotrowska-Niczyporuk et al. [11] who showed accelerated sulfur assimilation pathway under auxins and cytokinins treatment which led to increases in the synthesis of GSH in *A*. *obliquus* resulting in enhanced tolerance under Pb stress.

## Conclusions

We conclude that Cd has caused oxidative stress in *Trigonella* seedlings, and AsA-GSH cycle was not able to control the Cd induced damage which disturbed the redox status of the cell as manifested by decreased AsA/DHA and GSH/GSSG ratios. Supplementation of KN at low and medium doses up-regulated the enzymes of AsA-GSH cycle that maintains the redox status of cells, as evidenced by the increased content of AsA and GSH and ratios of AsA/DHA and GSH/GSSG which enhanced the tolerance of *Trigonella* seedlings under Cd stress.

## References

[1] Al-WailiN, SalomK, Al-GhamdiA, AnsariMJ. Antibiotic, pesticide, and microbial contaminants of honey: human health hazards. The scientific world Journal. 2012 Oct;2012. 10.1100/2012/930849.PMC347765923097637

[2] KumarA, ChauhanA, AroraS, TripathiA, AlghanemSM, KhanKA, et al. Chemical analysis of trace metal contamination in the air of industrial area of Gajraula (UP), India. Journal of King Saud University-Science. 2020 Jan 1;32(1):1106–10.

RETRACTED

[3] AltafR, AltafS, HussainM, ShahRU, UllahR, UllahMI, et al. Heavy metal accumulation by roadside vegetation and implications for pollution control. Plos one. 2021 May 13;16(5):e0249147. doi: 10.1371/journal.pone.0249147 33983956PMC8118294

[4] XinJP, MaS, ZhaoC, LiY, TianRN. Cadmium phytotoxicity, related physiological changes in Pontederia cordata: antioxidative, osmoregulatory substances, phytochelatins, photosynthesis, and chlorophyll fluorescence. Environmental Science and Pollution Research. 2020 Nov;27(33):41596–608. doi: 10.1007/s11356-020-10002-z 32691317

[5] BashriG, PrasadSM. Exogenous IAA differentially affects growth, oxidative stress and antioxidants system in Cd stressed *Trigonellafoenum-graecum* L. seedlings: Toxicity alleviation by up-regulation of ascorbate- glutathione cycle. Ecotoxicol. Environ. Saf. 2016; 132: 329–338. doi: 10.1016/j.ecoenv.2016.06.015 27344401

[6] MittlerR. Oxidative stress, antioxidants and stress tolerance. Trends Plant Sci. 2002; 7: 405–410. doi: 10.1016/s1360-1385(02)02312-9 12234732

[7] GillSS, TutejaN. Reactive oxygen species and antioxidant machinery in abiotic stress tolerance in crop plants. Plant Physiol Biochem. 2010; 48: 909–930. doi: 10.1016/j.plaphy.2010.08.016 20870416

[8] FoyerCH, NoctorG. Ascorbate and glutathione: the heart of the redox hub. Plant Physiol. 2011; 155: 2–18. doi: 10.1104/pp.110.167569 21205630PMC3075780

[9] KayaC, AshrafM, AlyemeniMN, AhmadP. The role of nitrate reductase in brassinosteroid-induced endogenous nitric oxide generation to improve cadmium stress tolerance of pepper plants by upregulating the ascorbate-glutathione cycle. Ecotoxicol. Environ. Saf. 2020; 196: 110483. doi: 10.1016/j.ecoenv.2020.110483 32247238

[10] ChauhanA, AbuAmarahBA, KumarA, VermaJS, GhramhHA, KhanKA, et al. Influence of gibberellic acid and different salt concentrations on germination percentage and physiological parameters of oat cultivars. Saudi journal of biological sciences. 2019 Sep 1;26(6):1298–304. doi: 10.1016/j.sjbs.2019.04.014 31516361PMC6733775

[11] Piotrowska-NiczyporukA, BajguzA, KotowskaU, Zambrzycka-SzelewaE, SienkiewiczA. Auxins and cytokinins regulate phytohormone homeostasis and thiol-mediated detoxification in the green alga *Acutodesmus obliquus* exposed to lead stress. Sci. Rep. 2020; 10(1): pp.1–14. doi: 10.1038/s41598-019-56847-4 32576894PMC7311453

[12] LiSM, ZhengHX, ZhangXS, SuiN. Cytokinins as central regulators during plant growth and stress response. Plant Cell Rep. 2020; 1–12. doi: 10.1007/s00299-020-02599-9 33025178

RETRACTED

[13] AnsariMJ, KumarR, SinghK, DhaliwalHS. Characterization and molecular mapping of EMS-induced brittle culm mutants of diploid wheat (*Triticum monococcum* L.). Euphytica. 2012 Jul;186(1):165–76.

[14] AnsariMJ, Al-GhamdiA, UsmaniS, KumarR, NuruA, SinghK, et al. Characterization and gene mapping of a brittle culm mutant of diploid wheat (*Triticum monococcum* L.) with irregular xylem vessels development. Acta physiologiae plantarum. (2013a) Aug 1;35(8):2407–19.

[15] AnsariMJ, Al-GhamdiA, KumarR, UsmaniS, Al-AttalY, NuruA, et al. Characterization and gene mapping of a chlorophyll-deficient mutant clm1 of *Triticum monococcum* L. Biologia plantarum. (2013b) Sep 1;57(3):442–8.

[16] AnsariMJ, KumarR, SinghK, DhaliwalHS. Characterization and molecular mapping of a soft glume mutant in diploid wheat (*Triticum monococcum* L.). Cereal Research Communications. 2014 Jun 1;42(2):209–17.

[17] SinghS, PrasadSM. Growth, photosynthesis and oxidative responses of *Solanum melongena* L. seedlings to cadmium stress mechanism of toxicity amelioration by kinetin. Sci. Hortic. 2014; 176: 1–10.

[18] AhangerMA, AzizU, SahliAA, AlyemeniMN, AhmadP. Combined kinetin and spermidine treatments ameliorate growth and photosynthetic inhibition in *Vigna angularis* by up-regulating antioxidant and nitrogen metabolism under cadmium stress. Biomolecules. 2020; 10(1): 147. doi: 10.3390/biom10010147 31963299PMC7022836

[19] IlyasN., AmjidM.W., SaleemM.A., KhanW., WattooF.M., RanaR.M., et al., 2020. Quantitative trait loci (QTL) mapping for physiological and biochemical attributes in a Pasban90/Frontana recombinant inbred lines (RILs) population of wheat (Triticum aestivum) under salt stress condition. *Saudi journal of biological sciences*, 27(1), pp.341–351. doi: 10.1016/j.sjbs.2019.10.003 31889856PMC6933172

[20] ShehzadM, ZhouZ, DittaA, KhanM, CaiX, XuY, et al. Identification and characterization of genes related to salt stress tolerance within segregation distortion regions of genetic map in F2 population of upland cotton. PloS one. 2021 Mar 26;16(3):e0247593. doi: 10.1371/journal.pone.0247593 33770112PMC7997035

[21] KhalofahA, KhanMI, ArifM, HussainA, UllahR, IrfanM, et al. Deep placement of nitrogen fertilizer improves yield, nitrogen use efficiency and economic returns of transplanted fine rice. Plos one. 2021 Feb 25;16(2):e0247529. doi: 10.1371/journal.pone.0247529 33630922PMC7906316

[22] GemrotováM, KulkarniMG, StirkWA, StrnadM. et al. Seedlings of medicinal plants treated with either a cytokinin antagonist (PI-55) or an inhibitor of cytokinin degradation (INCYDE) are protected against the negative effects of cadmium. Plant Growth Regul. 2013; 71: 137–145.

RETRACTED

[23] LichtenthalerHK. Chlorophylls and carotenoids: pigments of photosynthetic biomembranes. Methods Enzymol.1987; 148: 350–382.

[24] WilburKM, AndersonNG. Electrometric and colorimetric determination of carbonic anhydrase. J. Biol. Chem.1948; 176: 147–154. 18886152

[25] Kurra-HottaM, SatohK, KatohS. Relationship between photosynthesis and chlorophyll content during leaf senescence of rice seedlings. Plant Cell Physiol.1987; 28: 1321–1329.

[26] StrasserRJ, SrivastavaA, Tsimilli-MichaelM. The fluorescence transient as a tool to characterize and screen photosynthetic samples. In: YunusM., PathreU., MohantyP. (Eds.), Probing Photosynthesis: Mechanism, Regulation and Adaptation. Taylor and Francis, London, UK, 2000; pp. 443–480 (Chapter 25).

[27] VelikovaV, YordanovI, EdrevaA. Oxidative stress and some antioxidant systems in acid rain-treated bean plants: protective role of exogenous polyamines. Plant science. 2000 Feb 7;151(1):59–66.

[28] Thordal-ChristensenH, ZhangZ, WeiY, CollingeDB. Subcellular localization of H_2_O_2_ in plants: H_2_O_2_ accumulation in papillae and hypersensitive response during the barley-powdery mildew interaction. Plant J. 1997; 11: 1187–1194.

[29] NakanoY, AsadaK. Hydrogen peroxide is scavenged by ascorbate specific peroxidase in spinach chloroplasts. Plant Cell Physiol. 1981; 22: 867–880.

[30] SchaedleM, BasshamJA. Chloroplasts glutathione reductase. Plant Physiol. 1977; 59: 1011–1012. doi: 10.1104/pp.59.5.1011 16659940PMC543356

[31] GossettDR, MillhollonEP, LucasMC. Antioxidant response to NaCl stress in salt‐tolerant and salt‐sensitive cultivars of cotton. Crop science. 1994 May;34(3):706–14.

[32] BreheJE, BurchHB. Enzymatic assay for glutathione. Analytical biochemistry. 1976 Jul 1;74(1):189–97. doi: 10.1016/0003-2697(76)90323-7 962073

[33] ZhouM, GhnayaT, DaillyH, CuiG, VanpeeB, HanR, et al. The cytokinin trans-zeatineriboside increased resistance to heavy metals in the halophyte plant species *Kosteletzkyapenta carpos* in the absence but not in the presence of NaCl. Chemosphere. 2019; 233: 954–965. doi: 10.1016/j.chemosphere.2019.06.023 31340423

[34] AldesuquyH, BakaZ, MickkyB. Kinetin and spermine mediated induction of salt tolerance in wheat plants: Leaf area, photosynthesis and chloroplast ultrastructure of flag leaf at ear emergence. Egypt J Basic Appl Sci. 2014; 10.1016/j.ejbas.2014.03.002.

[35] YaronskayaE, VershilovskayaI, PoersY, AlawadyA, AverinaN, GrimmB. Cytokinin effects on tetrapyrrole biosynthesis and photosynthetic activity in barley seedlings. Planta. 2006; 224: 700–709. doi: 10.1007/s00425-006-0249-5 16506064

[36] PopovaLP, MaslenkovaLT, YordanovaRY, IvanovaAP, KrantevAP, SzalaiG, et al. Exogenous treatment with salicylic acid attenuates cadmium toxicity in pea seedlings. Plant Physiol Biochem.2009; 47: 224–31. doi: 10.1016/j.plaphy.2008.11.007 19091585

RETRACTED

[37] DurandTC, SergeantK, PlanchonS, CarpinS, LabelP, MorabitoD, et al. Acute metal stress *in Populus tremula* × *P. alba* (717-1B4 genotype): leaf and cambial proteome changes induced by cadmium (^2+^). Proteomics. 2010; 10: 349–368. doi: 10.1002/pmic.200900484 20148406

[38] ZhaoFJ, JiangRF, DunhamSJ, McGrathSP. Cadmium uptake, translocation and tolerance in the hyperaccumulator *Arabidopsis halleri*. New Phytol. 2006; 172: 646–654. doi: 10.1111/j.1469-8137.2006.01867.x 17096791

[39] FariduddinQ, AhmadA, HayatS. Response of *Vigna radiata* to foliar application of 28-homobrassinolide and kinetin. Biol Plant. 2004; 48: 465–468.

[40] PrasadSM, ZeeshanM. UV-B radiation and cadmium induced changes in growth, photosynthesis, and antioxidant enzymes of cyanobacterium *Plectonema boryanum*. Plant Biol.2005; 49: 229–236.

[41] Al-HakimiAMA. Modification of cadmium toxicity in pea seedlings by kinetin. Plant Soil Environ. 2007; 53: 129–135.

[42] Gonzalez-MendozaD, Espadasy GilF, SantamariaJM, Zapata-PerezO. Multiple effects of cadmium on the photosynthetic apparatus of *Avicennia germinans* L. as probed by OJIP chlorophyll fluorescence measurements. Z Naturfors C. 2007; 62:265–272. doi: 10.1515/znc-2007-3-418 17542495

[43] CortlevenA, NitschkeS, KlaumünzerM, et al. A novel protective function for cytokinin in the light stress response is mediated by the *Arabidopsis Histidine Kinase2* and *Arabidopsis Histidine Kinase3* receptors. Plant Physiol. 2014,164:1470–1483. doi: 10.1104/pp.113.224667 24424319PMC3938634

[44] TarakhovskayaER, KangEJ, KimKY, GarbaryDJ. Influence of phytohormones on morphology and chlorophyll a fluorescence parameters in embryos of Fucus vesiculosus L. (Phaeophyceae). Russ J Plant Physiol. 2013; 60(2): 176–183.

[45] LukatkinAS, GrachevaNV, GrishenkovaNN, DukhovskisPV, BrazaititeAA. Cytokinin-like growth regulators mitigate toxic action of zinc and nickel ions on maize seedlings. Russ. J Plant Physiol. 2007; 54:381–387.

[46] WuX, HeJ, DingH, ZhuZ, ChenJ, XuS, et al. Modulation of zinc-induced oxidative damage in *Solanum melongena* by 6-benzylaminopurine involves ascorbate–glutathione cycle metabolism. Environ Exp Bot., 2015; 116: 1–11.

